RETRACTED

# Nucleus pulposus cell senescence is alleviated by resveratrol through regulating the ROS/NF-κB pathway under high-magnitude compression

**DOI:** 10.1042/BSR20180670

**Published:** 2018-07-06

**Authors:** Yanhai Jiang, Guozhang Dong, Yeliang Song

**Affiliations:** Department of Orthopaedics, The Weihai Second Hospital Affiliated to Qingdao University, Weihai 264200, China

**Keywords:** cell senescence, compression, nucleus pulposus, resveratrol

## Abstract

Mechanical overloading is a risk factor of disc degeneration. Studies have demonstrated that resveratrol helps to maintain the disc cell’s healthy biology. The present study aims to investigate whether resveratrol can suppress mechanical overloading-induced nucleus pulposus (NP) cell senescence *in vitro* and the potential mechanism. The isolated rat NP cells were seeded in the decalcified bone matrix (DBM) and cultured under non-compression (control) and compression (20% deformation, 1.0 Hz, 6 h/day) for 5 days using the mechanically active bioreactor. The resveratrol (30 and 60 μM) was added into the culture medium of the compression group to investigate its protective effects against the NP cell senescence. NP cell senescence was evaluated by cell proliferation, cell cycle, senescence-associated β-galactosidase (SA-β-Gal) activity, telomerase (TE) activity, and gene expression of the senescence markers (p16 and p53). Additionally, the reactive oxygen species (ROS) content and activity of the NF-κB pathway were also analyzed. Compared with the non-compression group, the high-magnitude compression significantly promoted NP cell senescence, increased ROS generation and activity of the NF-κB pathway. However, resveratrol partly attenuated NP cell senescence, decreased ROS generation and activity of the NF-κB pathway in a concentration-dependent manner under mechanical compression. Resveratrol can alleviate mechanical overloading-induced NP cell senescence through regulating the ROS/NF-κB pathway. The present study provides that resveratrol may be a potential drug for retarding mechanical overloading-induced NP cell senescence.

## Introduction

Intervertebral disc (IVD) degeneration (IDD) is a fundamental structure that interspaces and connects the adjacent vertebral bones [1]. IDD often leads to instability, stenosis, and deformity of the spine motion segment, which ultimately causes some neurological symptoms [2]. Although disc degeneration is worldwide prevalent and causes a high socioeconomic burden [3], the accurate molecular mechanisms underlying the disc degeneration remain unclear. Current therapies, either conservative treatment or surgery treatment are mainly focussed on symptom relief but not the onset of disc degeneration.

RETRACTED

The IVD consists of three structurally integrated parts: the lamellar annulus fibrosis (AF), the gelatinous nucleus pulposus (NP), and the cartilaginous cartilage end plate (CEP) [4]. During disc degeneration, degenerative changes first occur in the disc NP region, which leads to decrease in NP cellular density and increase in NP matrix degradation [5,6]. Amongst these degenerative changes, disc NP cell senescence is a classical feature during disc degeneration and is often identified to be positively and closely correlated with disc degeneration grade [7–9].

As an inducing and initiating risk factor of disc degeneration, mechanical load often does harm to the healthy status of disc biology [10]. Moreover, a recent study has demonstrated that mechanical overloading accelerates disc NP cell senescence and inhibits NP matrix synthesis [11]. In line with this, an animal disc degeneration model induced by foreleg amputation also indicates that overloaded compression may contribute to the increased cellular senescence and the resulting disc degeneration [12–14]. It is well established that oxidative stress caused by reactive oxygen species (ROS) accumulation contributes to the cellular senescent-like cell function decline [15]. Furthermore, ROS content is also elevated in the degenerative human discs [16,17]. Importantly, excessive mechanical loading can increase the release of ROS from mitochondria in cartilage [18–20]. Based on the above statements, we deduce that inhibition of mechanical overloading-induced ROS accumulation may be effective in attenuating disc NP cell senescence.

Resveratrol, a natural phytoalexin that is found in plants including peanuts and grapes, is reported to have wide protective effects in different cell types, such as anti-inflammatory, anti-ageing, and cartilage protection [21–23]. However, whether it can attenuate mechanical overloading-induced NP cell senescence remains unknown, as well as the potential signaling transduction pathways. Therefore, in the present study, we mainly aimed to investigate the effects of resveratrol on disc NP cell senescence under mechanical overloading and the potential mechanisms in this regulatory process.

## Materials and methods

### NP cell isolation and scaffold pre-culture

Thirty-two Sprague–Dawley rats (male, 230–250 g, and 7–8 weeks old) were used according to the guidance of the Ethics Committee at the Weihai Second Hospital Affiliated to Qingdao University [SHNK(E) 2011-021]. Briefly, after the rats were killed by inhaling excessive carbon dioxide, the lumbar discs (L1–L5) were separated and the central gelatinous NP tissue was removed using the No. 11 surgical blade. Thereafter, NP samples were subjected to the sequential enzymatic digestion with 0.25% trypsin (Gibco, U.S.A.) for 5 min and 0.25% type I collagenase (Sigma, U.S.A.) for 10–15 min, as described in a recent study [24]. Then, NP cell pellets were collected by centrifugation and re-suspended in DMEM/F12 medium (HyClone, U.S.A.) containing 10% (v/v) FBS (Gibco), and 1% (v/v) penicillin–streptomycin (Gibco, U.S.A.) under the standard conditions (37°C, 21% O_2_ and 5% CO_2_). The culture medium was refreshed every 3 days. Because subcultivation can lead to cellular senescence, passage 2 (P2) NP cells were first suspended in the collagen solution (1 mg/ml, Shengyou, China) and then were seeded into the prepared bovine decalcified bone matrix (DBM, 10 × 10 × 5 mm, 1 × 10^7^ cells per DBM) scaffold as previously described [25,26]. Before dynamic compression, NP cells seeded in DBM scaffolds were pre-cultured for 2 days under the standard conditions (37°C, 21% O_2_ and 5% CO_2_).

RETRACTED

### Grouping and dynamic compression application

To study the effects of resveratrol on high magnitude, compression-induced NP cell senescence, four groups were designed: control group (non-compression), compression (20% compressive deformation) group, compression (20% compressive deformation) + resveratrol (30 μM) group, and compression (20% compressive deformation) + resveratrol (60 μM) group. The concentration of resveratrol was determined according to a recent study [27]. Because the NP cells were seeded into the DBM scaffolds, we could not directly calculate how much mechanical magnitude was experienced by NP cells, and the compression magnitude was just reflected and described according to the compressive deformation of the DBM construct. The dynamic compression was applied by a mechanically active bioreactor. The 20% deformation of compressive magnitude (at a frequency of 1.0 Hz for 6 h once per day) was defined according to the disc height alteration in a day (20–25%). NP cells seeded in the DBM scaffolds were cultured and dynamically compressed for 5 days in the mechanically active bioreactor. The resveratrol was added along with the culture medium of the compression group to study its effects on NP cell senescence.

### Cell proliferation assay

After dynamic compression, NP cells seeded in the DBM scaffold were collected by digestion with 0.05% trypsin and 0.1% collagenase for 40–60 s. Then, NP cells (3 × 10^3^ cells per group) were seeded in the 96-well plate and NP cell proliferation was detected at 6, 24, and 48 h with a cell counting kit-8 (CCK-8, Beyotime, China) and a Click-iT EdU microplate assay kit (Invitrogen, U.S.A.) according to the manufacturer’s instructions. The NP cell proliferation rate was expressed as optical density value at 450 nm (OD450) wavelength and the relative fluorescence units (RFU) detected at 490/585 nm (excitation/emission wavelength), respectively.

RETRACTED

### Senescence-associated β-galactosidase activity

NP cells (1 × 10^4^ per group) collected from the DBM scaffolds were first subjected to adherent culture for 5–6 h. Then, senescence-associated β-galactosidase (SA-β-Gal) staining was performed according to the manufacturer’s instructions (senescence β-galactosidase staining kit, Beyotime, China). The SA-β-Gal staining-positive NP cells were observed under a light microscope (Olympus BX51) and quantitated using the ImagePro Plus software (version 5.1, Media Cybernetics, Inc.).

### Cell cycle analysis

NP cells collected from the DBM scaffolds were harvested and washed with phosphate buffer solution (PBS), followed by fixation with 75% ethanol overnight at 4°C. Then, they were incubated with Propidium Iodide dye (50 μg/ml, Beyotime, China) and RNase A (100 μg/ml, Beyotime, China) for 30 min. Finally, the prepared NP cells were subjected to a flow cytometry machine (FACS Aria; BD Company), and the cell cycle phases of G_0_/G_1_, G_2_/M, and S were analyzed by multicycle software (PHENIX Company, Japan).

### Telomerase activity

First, NP cells were collected from the DBM scaffold as described above after compression. Then, NP cell pellets were incubated with RIPA lysis buffer (Beyotime, China) for 15 min. Then, equal volume of supernatant in each group was used to detect telomerase (TE) activity (IU/l) according to the manufacturer’s instructions (TE ELISA kit, Mlbio, China).

### ROS content measurement

After NP cells seeded in the DBM scaffold were incubated with the fluorescent probe DCFH-DA (10 μM, Nanjing Jiancheng Bioengineering Institute, China) in a humidified atmosphere for 30 min, they were collected as described above and washed with PBS for two times. Finally, NP cells (1 × 10^5^ per group) were used to analyze intracellular ROS generation that was expressed as RFU at an excitation/emission wavelength of 490/585 nm.

### Real-time PCR analysis

Gene expression of senescence markers (p16 and p53) was analyzed by real-time PCR. Briefly, after DBM scaffolds were cut into small pieces, total RNA was extracted using the Tripure Isolation Reagent (Roche, Switzerland) and synthesized into cDNA using the First Strand cDNA Synthesis Kit (Roche, Switzerland). Then, a reaction mixture containing cDNA, SYBR Green Mix (TOYOBO, Japan), and primers (Table 1) was subjected to the PCR. The PCR parameters were: 3 min at 95°C, followed by 40 amplification cycles of 20 s at 95°C, 10 s at 56°C, and 10 s at 72°C. β-actin was used as an internal reference and the gene expression was calculated according to the method of 2^−ΔΔ*C*^_t_.

RETRACTED

**Table 1:** Primers of target genes

Gene	Forward (5′–3′)	Reverse (5′–3′)
*β-actin*	CCGCGAGTACAACCTTCTTG	TGACCCATACCCACCATCAC
*P53*	CCTTAAGATCCGTGGGCGT	GCTAGCAGTTTGGGCTTTCC
*P16*	TACCCCGATACAGGTGATGA	TACCGCAAATACCGCACGA

### Western blot analysis

The protein expression of p16, p53, NF-κB p65, and p-NF-κB p65 was analyzed by Western blot assay. Briefly, after DBM scaffolds were cut into small pieces, total protein was extracted using RIPA solution (Beyotime, China). Then, equal protein samples in each group were subjected to SDS/PAGE system and transferred on to PVDF membranes. Then, the PVDF membranes were incubated with primary antibodies (p16: Novus, NBP2-37740; p53: Proteintech, 10442-1-AP; NF-κB p65: Beyotime, AV365; p-NF-κB p65: Beyotime, AV371; β-actin, Proteintech, 60008-1-Ig; all diluted 1:1000) at 4°C overnight, followed by incubation with the corresponding HRP-conjugated secondary antibodies (ZSGB-BIO, China, diluted 1:2000) at 37°C for 2 h. After protein bands on the PVDF membrane were developed using a SuperSignal West Pico Trial Kit (Thermo, U.S.A.); protein expression normalized to β-actin was analyzed using the ImageJ software (National Institutes of Health, U.S.A.).

### Statistical analysis

In the current study, all numerical data were expressed as the means ± S.D., and each experiment was performed in triplicate. After the homogeneity test for variance, intergroup comparisons were performed via ANOVA using SPSS 13.0 software, and the post hoc test was determined by the LSD test. A significant difference was indicated when the *P*-value <0.05.

## Results

### Cell proliferation

Senescent cells often have a low potency of cellular proliferation [28]. Here, NP cell proliferation was evaluated by CCK-8 assay (Figure 1A) and EdU incorporation assay (Figure 1B). Results showed that the value of OD450 and RFU (490/585 nm) in the compression group (20% deformation) was significantly decreased compared with the control (non-compression) group. However, the addition of resveratrol partly attenuated the effects of this high-magnitude compression on NP cell proliferation, with a higher resveratrol concentration (60 μM) group exhibited more obvious protective effects on cell proliferation than a lower resveratrol concentration (30 μM).

**Figure 1:** Resveratrol stimulated NP cell proliferation in a dose-dependant manner (**A**) Cell proliferation evaluated by CCK-8 assay. (**B**) Cell proliferation evaluated by EdU incorporation assay. Data are expressed as mean ± S.D. (*n*=3). ^#^ indicates a statistical difference compared with the control group. * indicates a statistical difference (*P*<0.05) between two groups.

RETRACTED

### SA-β-Gal activity

SA-β-Gal staining is a commonly used parameter for identifying senescent cells because they often have increased SA-β-Gal activity [29]. Results showed that the percentage of SA-β-Gal staining-positive NP cells in the compression group (20% deformation) is much higher than in the control group (non-compression), whereas the resveratrol partly decreased the percentage of SA-β-Gal staining-positive NP cells under mechanical compression in a concentration-dependent manner (Figure 2).

**Figure 2:** Resveratrol decreased SA-β-Gal activity of NP cells in a dose-dependent manner Magnification: 200×; scale = 100 μM; *n*=3. Data are expressed as mean ± S.D. ^#^ indicates a statistical difference compared with the control group. * indicates a statistical difference (*P*<0.05) between two groups.

### Cell cycle

Cell cycle analysis is another parameter for evaluating cellular senescence. It has been well established that senescent cells are often arrested in the phase of G_0_/G_1_ [30]. Our results showed that NP cells in the compression group (20% deformation) had a significantly increased G_0_/G_1_ phase fraction and a significantly decreased S phase fraction compared with the control group (non-compression). Further analysis showed that the addition of resveratrol partly attenuated the effects of this high-magnitude compression on G_0_/G_1_ phase and S phase fraction, with a higher resveratrol concentration (60 μM) exhibited more obvious effects than a lower resveratrol concentration (30 μM) (Figure 3).

**Figure 3:** Resveratrol attenuated cell cycle arrest of NP cells in a dose-dependent manner The histogram shows the cell fraction proportion of each cell cycle (G_0_/G_1_, S, and G_2_/M) amongst these groups.

### TE activity

TE activity is also often used in previous studies to evaluate cellular senescence [31]. A decreased TE activity reflects an aggravation of cellular senescence. Results showed that the TE activity in the compression group (20% deformation) obviously decreased compared with the control group (non-compression). Resveratrol partly increased TE activity under this high-magnitude compression in a concentration-dependent manner (Figure 4).

**Figure 4:** Resveratrol decreased TE activity of NP cells in a dose-dependent manner Data are expressed as mean ± S.D. (*n*=3). ^#^ indicates a statistical difference compared with the control group. * indicates a statistical difference (*P*<0.05) between two groups.

### Gene expression analysis

The p53-p21-pRb pathway and the p16-pRb pathway are two theoretical signaling transduction mechanisms responsible for cellular senescence [32]. Hence, p53 and p16 are often used as classical senescence markers. Results showed that gene expression of these two senescence markers (p16 and p53) in the compression group (20% deformation) were significantly up-regulated compared with the control group (non-compression), and that the addition of resveratrol partly suppressed their gene expression levels in a concentration-dependent manner (Figure 5).

RETRACTED

**Figure 5:** Resveratrol down-regulated senescence markers expression of NP cells in a dose-dependent manner (**A**) Gene expression of p16 and p53. (**B**) Protein expression of p16 and p53. Data are expressed as mean ± S.D. (*n*=3). ^#^ indicates a statistical difference compared with the control group. * indicates a statistical difference (*P*<0.05) between two groups.

### Intracellular ROS accumulation and activity of NF-κB pathway

Oxidative stress damage caused by intracellular ROS accumulation largely contributes to the cellular senescence [15]. In the present study, we analyzed ROS content and the activity of its downstream NF-κB pathway. Results showed that ROS content in the compression group (20% deformation) was much higher than in the control group (non-compression), whereas the addition of resveratrol partly decreased the generation of intracellular ROS in a concentration-dependent manner (Figure 6A). Similarly, we found that activity of the NF-κB pathway showed a similar trend to the ROS generation amongst these groups (Figure 6B).

**Figure 6:** Resveratrol decreased intracellular ROS content and NF-κB pathway activity in NP cells (**A**) ROS content measurement. (**B**) Western blotting analysis of activation of the NF-κB pathway. Data are expressed as mean ± S.D. (*n*=3). ^#^ indicates a statistical difference compared with the control group. * indicates a statistical difference (*P*<0.05) between two groups.

## Discussion

Disc degeneration-induced leg and low back pain are the leading causes of physical disability [33]. Excessive or inappropriate mechanical loading is a well-known contributing factor of disc degeneration [34]. Previous studies have indicated that excessive mechanical loading can lead to disc NP cell senescence [12–14]. In the current study, we confirmed that high-magnitude compression significantly promoted NP cell senescence and demonstrated that resveratrol partly attenuated mechanical overloading-induced NP cell senescence in a concentration-dependent manner. The present study provides potential therapeutic effects of resveratrol on mechanical overloading-induced disc degeneration.

Due to the implication of cellular senescence during disc degeneration, a comprehensive understanding and identification of senescent cells are necessary. Conventionally, senescent cells have suppressed cell proliferation, increased SA-β-Gal activity, promoted G_0_/G_1_ cell cycle arrest, decreased TE activity, and up-regulated senescence marker’s expression [29–32]. Therefore, in the present study, we evaluated NP cell senescence by cell proliferation assay, SA-β-staining, cell cycle, and TE activity. The results showed that this high-magnitude compression significantly suppressed NP cell proliferation, increased SA-β-Gal activity and G_0_/G_1_ phase fraction, and decreased TE activity, indicating that this high magnitude can promote NP cell senescence. This is in line with previous studies [13,14]. However, the addition of resveratrol partly attenuated the change of all these parameters, suggesting that resveratrol may alleviate NP cell senescence under mechanical overloading to some extent.

RETRACTED

Two mechanisms are responsible for cellular senescence: the telomere-based p53-p21-pRB pathway representing replicative senescence (RS) and the stress-based p16-pRB pathway representing stress-induced premature senescence (SIPS) [35]. A previous study has demonstrated that either p16 or p53, or both of them are up-regulated in the degenerative disc tissue [36]. In the present study, we found that this high-magnitude compression up-regulated expression of both p16 and p53 compared with the non-compression group, indicating that mechanical overloading can accelerate NP cell senescence through the RS and SIPS pathway. However, the addition of resveratrol partly down-regulated expression of these two senescence markers (p16 and p53) in a concentration-dependent manner, suggesting again that resveratrol can suppress mechanical overloading-induced NP cell senescence. In line with this, a recent study has also demonstrated that resveratrol can activate sirt1 and then play some protective effects, such as increasing NP cell proliferation, suppressing NP cell apoptosis, and enhancing NP matrix anabolism [37].

Based on the free-radical theory of ageing, oxidative stress caused by ROS accumulation is able to promote cellular senescence in many cell types [15]. Numerous degenerative disorders, such as osteoarthritis and neurodegenerative disease, are correlated with oxidative stress [38,39]. In the degenerative human discs, ROS generation is also elevated and is proved to be involved in age-related disc degeneration [16,17]. In the present study, we found that this high-magnitude compression significantly increased ROS generation compared with the non-compression group. This is in line with the study on cartilage and our own previous experience [20]. A recent study has shown that ROS generation is positively correlated with NP cell senescence under mechanical compression [24]. In the present study, the addition of resveratrol suppressed ROS generation under the mechanical compression in a concentration-dependent manner. ROS generation is a common step in NF-κB activation that participates in cell apoptosis and cell proliferation [40]. In the present study, activity of the NF-κB pathway exhibited similar trend to its upstream regulator ROS. Collectively, these results indicate that resveratrol may alleviate NP cell senescence under mechanical compression through regulating the ROS-/NF-κB pathway.

RETRACTED

The present study also has several limitations. First, NP cells were scaffold-cultured under normoxic condition. This differs from the physiological conditions in which NP cells are embraced by the native extracellular matrix under hypoxic condition. Second, we did not verify these results in an *in vivo* animal model. If possible, we will develop a kind of device that can accurately apply dynamic compression to IVD to perform similar experiments using an *in vivo* animal model in the future. Third, the rat NP tissue contains lots of notochordal cells which disappear in the discs NP tissue of adult human. Though there are not any specific markers to differentiate NP cells from notochordal cells, their existence may bring inference to the actual results under mechanical compression and limit the strength in reflecting actual pathological phenomenon of disc degeneration in adult human.

Based on our results, we can draw the conclusion that resveratrol can alleviate mechanical overloading-induced NP cell senescence and that the ROS/NF-κB pathway may participate in this regulatory process. The present study, for the first time, sheds light on the protective effects of resveratrol against mechanical overloading-induced NP cell senescence.

## Abbreviations

CCK-8: cell counting kit-8
DBM: decalcified bone matrix
IDD: intervertebral disc degeneration
IVD: intervertebral disc
NP: nucleus pulposus
OD450: optical density value at 450 nm
PBS: phosphate buffer solution
RFU: relative fluorescence unit
ROS: reactive oxygen species
RS: replicative senescence
SA-β-Gal: senescence-associated β-galactosidase
SIPS: stress-induced premature senescence
TE: telomerase
